# Age at last birth and risk of developing epithelial ovarian cancer: a meta-analysis

**DOI:** 10.1042/BSR20182035

**Published:** 2019-09-13

**Authors:** Yanjun Wu, Wenjun Sun, Xueling Xin, Weijing Wang, Dongfeng Zhang

**Affiliations:** Department of Epidemiology and Health Statistics, the College of Public Health of Qingdao University, Qingdao, Shandong Province, People’s Republic of China

**Keywords:** age at last birth, ALB, epidemiology studies, epithelial ovarian cancer, meta-analysis

## Abstract

**Background:** Many epidemiologic studies have explored the association between age at last birth (ALB) and the risk of epithelial ovarian cancer, but the results remain controversial. **Methods:** A literature search was performed in PubMed, Web of Science, China National Knowledge Infrastructure (CNKI) and WanFang Med Online for relevant articles published up to April 2019. Pooled relative risks (RRs) with 95% confidence intervals (CIs) were calculated using a random-effect model. Dose–response relationship was assessed by restricted cubic spline model. **Results:** Thirteen articles with 19,959 cases and 2,451,071 participants were included in our meta-analysis, and we found that ALB was negatively associated with epithelial ovarian cancer. The pooled RR (95% CI) of epithelial ovarian cancer for the highest versus the lowest stratification of ALB was 0.77 (0.65–0.91). Furthermore, significantly negative associations were shown in case–control studies (RR: 0.73; 95% CI: 0.60–0.88), studies conducted in North America (RR: 0.71; 95% CI: 0.60–0.84), studies with adjustment for parity (RR: 0.76; 95%CI: 0.63–0.93), studies with adjustment for tubal ligation (RR: 0.74; 95% CI: 0.58–0.94), in the subgroup analysis. In dose–response analysis, the risk of epithelial ovarian cancer decreased nonlinearly with the increase of ALB, and the negative results become significant when ALB was 22.5 years old. **Conclusion:** This meta-analysis suggested that ALB was negatively associated with the risk of epithelial ovarian cancer. The risk of epithelial ovarian cancer decreased gradually with the ALB for women.

## Introduction

Epithelial ovarian cancer is a gynecologic malignancy with fairly high mortality. For most patients with epithelial ovarian cancer, they are diagnosed in advanced stages and have a poor prognosis [1]. According to cell histology, epithelial ovarian cancer is classified into four main subtypes: serous tumor (70–80%), clear cell tumor (5–10%), endometrioid tumor (10%) and mucinous tumor (3–4%) [1,2]. The menstrual, reproductive and hormonal factors are closely associated with the risk of developing epithelial ovarian cancer [3–8], and the role of some of these factors are now well investigated. Factors connected with a reduced risk of epithelial ovarian cancer include the use of oral contraceptive (OC), high parity, breastfeeding and a history of tubal ligation [7,9–12]. In the other hand, endometriosis, the use of menopausal hormone and later menopause are risk factors for epithelial ovarian cancer [13–15].

Age at last birth (ALB) plays a vital role in the pathogenesis of gynecological cancer, which maybe because of the prenatal hormone changes [16]. Study has found that a later ALB is associated with a lower risk of endometrial cancer [17]. However, the association between ALB and the risk of epithelial ovarian cancer is still controversial. Numerous epidemiological studies have been done to explore the association between ALB and the risk of epithelial ovarian cancer [3,18–29]. Among these studies, eight studies [18–20,22–24,26,29] showed no apparent association between ALB and epithelial ovarian cancer; four [21,25,27,28] showed a negative association; and one [3] showed a positive association. Thus, we conducted this meta-analysis to explore the association between ALB and risk of epithelial ovarian cancer systematically.

## Materials and methods

Preferred Reporting Items for Systematic reviews and Meta-Analyses (PRISMA) guidelines were consulted in this analysis [30].

### Literature search strategy

All relevant studies (up to April 2019) were identified by a comprehensive search in PubMed, Web of Science, Chinese National Knowledge Infrastructure (CNKI) and WanFang Med Online. Search terms included ‘age at last birth’ (or ‘age at last delivery’ or ‘age at last pregnancy’ or ‘age at last child’ or ‘age at last childbirth’ or ‘age at last full-term pregnancy’) and ‘ovarian cancer’ (or ‘oophoroma’ or ‘carcinoma of the ovary’ or ‘ovarian neoplasm’ or ‘ovarian tumor’). We also manually searched the relevant references within included studies to find eligible articles. The detailed steps of the literature selection are shown in Figure 1.

**Figure 1:** Flow chart of the selection of studies included in the meta-analysis

### Inclusion criteria

Two investigators (Yanjun Wu and Wenjun Sun) checked carefully all identified articles. If the article met the following criteria, it would be included in our meta-analysis. (1) a case–control or cohort study was published as an original study; (2) the exposure of interest was ALB; (3) the outcome of interest was epithelial ovarian cancer; (4) There was reported effect size (relative risk (RR) or odds ratio (OR) or hazard ratio (HR) or incidence rate ratio (IRR)) and 95% confidence interval (CI) for the association between ALB and epithelial ovarian cancer; (5) We selected the most recent study, if data from the same population were used in multiple articles.

### Data extraction

From each eligible article, we extracted the first author’s name, country where the study was conducted, publication year, the type of study design, the follow-up duration of cohort study, age range or mean age at baseline. We also extracted the number of cases and participants, the information about ALB, RRs (we presented all results as RR for simplicity) with their 95% CIs for each stratification of ALB, as well as adjusted factors.

### Statistical analysis

The lowest stratification of ALB was considered as the reference category in the majority of studies. When the reference category was not the lowest stratification of ALB [21,23,26], the method proposed by Hamling et al. [31] was used to convert risk estimates. In article [29] that only reported ‘floating absolute risk’ CIs, conventional CIs should be calculated by using the approach of Easton et al. [32]. For articles [27,29] that only reported on the association between ALB and epithelial ovarian cancer split by subgroup (e.g. menopausal status or tumor subtype), a random-effect model (REM) was first used to generate an overall result. Then a pooled measure was calculated as the inverse variance-weighted mean of the logarithm of RR with corresponding 95% CI to assess the strength of association between ALB and the risk of epithelial ovarian cancer. The *I^2^* of Higgins and Thompson was adopted to assess the heterogeneity among studies, and *I^2^* values of 0, 25, 50 and 75% represent no, low, moderate and high heterogeneity [33]. If *I^2^* < 50%, the fixed-effect model (FEM) would be used to combine study-specific RRs (95% CIs), otherwise, the REM which considers both within-study and between-study variation would be used (*I^2^* ≥ 50%) [34,35]. Meta-regression was used to explore the important potential covariates that might exert substantial impacts on between-study heterogeneity [36]. Subgroup analyses were performed by continent, the type of study design, whether or not the results were adjusted for parity, the use of OC and tubal ligation. Leave-One-Out sensitivity analysis was performed to evaluate the pivotal studies that have substantial impacts on between-study heterogeneity [37]. The influence analysis was performed to assess whether the result could have been affected obviously by a single study. Publication bias was evaluated using the Egger’s test and funnel plot [38].

For dose–response analysis, a two-stage random-effects dose–response meta-analysis [39] was performed. In the first stage, a restricted cubic spline model with three knots at the 25th, 50th and 75th centiles [40] of the levels of ALB was estimated using generalized least square regression, taking into account the correlation within each set of published RRs [41]. Then the study-specific estimates were combined using the restricted maximum likelihood method in a multivariate random-effects meta-analysis [42]. A *P-*value for nonlinearity was calculated by testing the null hypothesis that the coefficient of the second spline is equal to 0.

All statistical analyses were performed with Stata version 15.0 (Stata Corp., College Station, TX, U.S.A.). All reported probabilities (*P*-values) were two-sided, and *P*-values less than 0.05 were considered statistically significant.

## Results

### Literature search and characteristic of included studies

Using our search strategy mentioned in ‘material and method’, we identified 334 articles in total. There were 168 articles from PubMed, 251 articles from Web of Science, 10 articles from Wan Fang Med Online and 4 articles from reference list of included articles. We excluded 286 articles after reviewing the title and abstract, and we further excluded 35 articles in the step of full-text article reviewing. Among these 35 articles, the outcome of 4 articles [43–46] was ovarian cancer (not restricted to epithelial ovarian cancer), the outcome of one article was ovarian cancer survival [47], two articles [48,49] had the same population, 16 articles failed to evaluate the association between ALB and epithelial ovarian cancer and 12 articles did not report RRs and 95% CIs for the association of interest. Ultimately, thirteen [3,18–29] articles were included in our meta-analysis. The detailed steps of the article selection were shown in Figure 1. In these included articles, seven studies [19–24,27] were conducted in North America, five [3,18,26,28,29] in Europe and one [25] in Oceania. With regard to the type of study design, ten articles [3,19–22,24–28] were case–control studies and three [18,23,29] were cohort studies. The characteristics of the included studies are shown in Table 1.

**Table 1:** Characteristics of the included studies for ALB with risk of the epithelial ovarian cancer

First author	Country (year)	Age range or Mean age (Case/control)	Study design (years of follow up)	Exposure (ALB)	Case	Participants	RR(95% CI)	Adjustment for covariates
Gaitskell	U.K. (2018)	56.1	Cohort (14.6)	<25	1002	1144762	1	Age, region, tubal ligation, hysterectomy, family history of breast cancer, the use of OC, use of menopausal hormones, BMI, smoking, SES, parity.
				25–29	2043		0.96 (0.89–1.04)	
				≥30	1823		0.93 (0.85–1.01)	
Sköld	Nordic (2018)	19–85	Case–control	<25	1455	118821	1	Parity.
				25–29	3454		0.85 (0.80–0.91)	
				30–39	5556		0.76 (0.71–0.82)	
				≥40	492		0.64 (0.56–0.72)	
Moorman	America (2008)	20–74	Case–control	<25	190	1543	1	Age, race, family history of breast or ovarian cancer, age at menarche, tubal ligation, parity, infertility, BMI, the use of OC, age at last OC use, age at first pregnancy, years since first pregnancy, years since last pregnancy, breastfeeding.
				25–29	248		0.87 (0.65–1.18)	
				30–34	190		0.67 (0.50–0.89)	
				≥35	79		0.54 (0.38–0.77)	
Soegaard	Denmark (2007)	35–79	Case–control	<25	100	1927	1	Age, pregnancy, parity, the use of OC.
				25–29	147		0.66 (0.48–0.91)	
				≥30	222		0.68 (0.45–1.01)	
Whiteman	Australia (2003)	18–79	Case–control	<25	117	1343	1	Parity, the use of OC, tubal ligation, hysterectomy, smoking, alcohol use, time since last birth.
				25–29	212		0.75 (0.52–1.10)	
				30–34	171		0.56 (0.37–0.84)	
				≥35	120		0.57 (0.36–0.90)	
Tung	America (2003)	18+	Case–control	<28	NA	NA	1	Age, ethnicity, study site, education, the use of OC, tubal ligation.
				28–30			1.10 (0.70–1.60)	
				31–34			1.00 (0.70–1.40)	
				>34			0.90 (0.60–1.30)	
Vachon	America (2002)	56–81	Cohort (13)	≤29	66	31377	1	Hysterectomy, physical activity, waist-to-hip ratio, parity.
				30–34	40		0.76 (0.51–1.13)	
				≥35	48		0.97 (0.54–1.74)	
Titus-Ernstoff	America (2001)	20–74	Case–control	<25	69	795	1	Age, state, parity.
				25–29	119		0.62 (0.40–0.99)	
				30–34	110		0.62 (0.34–1.13)	
				≥35	80		0.62 (0.33–1.19)	
Cooper	America (1999)	18–79	Case–control	≤25	199	4060	1	Age, study, race, history of breast or ovarian cancer, the use of OC, tubal ligation, parity.
				26–30	201		0.64 (0.43–0.96)	
				≥31	228		0.71 (0.53–0.96)	
Salazar-Martinez	Mexico (1999)	52.8/54.6	Case–control	≤25	36	752	1	Age, anovulatory index, smoking, diabetes mellitus, hypertension, physical activity, menopausal status, body build index.
				26–35	28		0.65 (0.34–1.20)	
				≥36	20		0.87 (0.40–1.80)	
Godard	Canada (1998)	20–84	Case–control	17–29	NA	NA	1	NA.
				30–44			0.63 (0.34–1.15)	
Albrektsen	Norway (1996)	20–56	Cohort (16.4)	<25	218	1145076	1	Age, birth-cohort, parity, age at first birth, time since last birth.
				25–29	416		0.93 (0.77–1.12)	
				30–34	256		0.84 (0.66–1.08)	
				≥35	81		0.77 (0.54–1.11)	
Tavani	Italy (1993)	15–44	Case–control	<25	23	615	1	Age, education, family history, parity, number of abortions, the use of OC.
				25–29	48		1.30 (0.70–2.40)	
				≥30	52		2.40 (1.30–4.50)	

Abbreviations: BMI, body mass index; NA, not available; SES, socioeconomic status.

### Overall association between ALB and epithelial ovarian cancer

Thirteen articles [3,18–29] involving 19,959 cases and 2,451,071 participants were included to evaluate the association between ALB and epithelial ovarian cancer. Among these studies, eight studies [18–20,22–24,26,29] showed no apparent association between ALB and epithelial ovarian cancer; four [21,25,27,28] showed a negative association; and one [3] showed a positive association. The pooled RR of epithelial ovarian cancer for the highest versus the lowest stratification of ALB was 0.77 (95% CI: 0.65–0.91; *I^2^* = 73.90%, *P*_for heterogeneity_<0.001). The detailed results are shown in Figure 2.

**Figure 2:** Forest plot of ALB and the risk of epithelial ovarian cancer The size of gray box is positively proportional to the weight assigned to each study, and horizontal lines represent the 95% CIs. The RR (95%CI) in every article is the RR (95% CI) of epithelial ovarian cancer for the highest versus the lowest stratification of ALB.

In dose–response analysis, data from nine studies [3,20–23,25–28] were used and a nonlinear association was found (*P*_nonlinearity_=0.004) between ALB and risk of epithelial ovarian cancer. The risk of epithelial ovarian cancer decreased gradually with the ALB, and the results become significant when ALB was 22.5 years old. The RRs (95% CIs) of epithelial ovarian cancer risk for the 25th, 50th and 75th centiles of the levels of ALB were 0.99 (0.99–0.99), 0.95 (0.94–0.96) and 0.88 (0.86–0.90) for 22.5, 27.5 and 32.5 years old, respectively. The detail results are shown in Figure 3.

**Figure 3:** The dose–response analysis between ALB and the risk of epithelial ovarian cancer with restricted cubic splines in a multivariate random-effects dose–response model The solid line and the long dash line represent the estimated RRs and its 95% CIs. Short dash line represents the linear relationship.

Data from five studies [22,24,26,28,29] were used to explore the association between ALB and the histologic subtypes of epithelial ovarian tumor. The pooled RR (95%CI) for the highest versus the lowest stratification of ALB was 0.80 (0.62–1.03) for serous tumors, 0.91 (0.77–1.07) for mucinous tumors, 0.72 (0.42–1.24) for endometrioid tumors and 0.83 (0.63–1.09) for clear cell tumors. The characteristics of the included studies and the detailed results are shown in Table 2.

**Table 2:** RRs and 95% CIs for the association between ALB and risk of the major epithelial ovarian cancer subtypes

Author (year)	Exposure (ALB)	Histologic subtypes of epithelial ovarian cancer					
		Serous		Mucinous		Endometrioid	Clear cell
Gaitskell (2018)	≥30/<25	0.94 (0.85–1.04)		0.91 (0.74–1.12)		0.96 (0.74–1.24)	0.78 (0.56–1.08)
Titus-Ernstoff (2001)	≥30/<30	Borderline	Invasive	1.10 (0.60–2.00)			
		0.80 (0.40–1.60)	1.00 (0.70–1.50)				
Soegaard (2007)	≥30/<25	0.64 (0.39–1.04)		0.74 (0.25–2.18)		0.71 (0.27–1.89)	
Sköld (2018)	≥40/<25	0.58 (0.48–0.70)		0.93 (0.65–1.34)		0.39 (0.24–0.65)	1.01 (0.57–1.79)
Tung (2003)	>34/<28	Borderline	Invasive	Borderline	Invasive	1.10 (0.40–2.70)	0.80 (0.30–2.00)
		0.50 (0.20–1.30)	1.20 (0.70–1.90)	0.60 (0.20–1.50)	0.70 (0.20–2.20)		
Pooled RR (95% CI)	The highest versus the lowest stratification	0.80 (0.62–1.03) *I^2^* = 75.70%, *P*<0.001		0.91 (0.77–1.07) *I^2^* = 0.00%, *P*=0.927		0.72 (0.42–1.24) *I^2^* = 71.10%, *P*=0.016	0.83 (0.63–1.09) *I^2^* = 0.00%, *P*=0.743

### Subgroup analysis

In the subgroup analysis by continent where the study was conducted, the pooled RRs (95% CIs) were 0.71 (0.60–0.84) and 0.86 (0.65–1.14) for the studies conducted in North America and Europe, respectively. In the subgroup analysis by study design, the pooled RRs (95% CIs) for case–control and cohort studies were 0.73 (0.60–0.88) and 0.92 (0.85–1.00), separately. According to whether the results were adjusted for parity or not, the pooled RRs (95% CIs) were 0.76 (0.63–0.93) and 0.82 (0.61–1.11) for studies with adjustment and without, respectively. According to whether the results were adjusted for the use of OC or not, the pooled RRs (95% CIs) for studies with adjustment and without were 0.81 (0.63–1.03) and 0.66 (0.59–0.74), severally. In the subgroup analysis of whether the results were adjusted for the tubal ligation or not, the pooled RRs (95% CIs) for studies with adjustment and without were 0.74 (0.58–0.94) and 0.81 (0.62–1.04), respectively. Detailed results of subgroup analysis are shown in Table 3.

**Table 3:** Summary of subgroup results for association of ALB with risk of the epithelial ovarian cancer

Stratification	Number of studies	RR (95% CI)	*I^2^*,%	*P*_for heterogeneity_
All studies	13	0.77 (0.65–0.91)	73.90%	<0.001
Continent where the study was conducted				
North America	7	0.71 (0.60–0.84)	0.00%	0.488
Oceania	1	0.57 (0.36–0.90)		
Europe	5	0.86 (0.65–1.14)	88.70%	<0.001
The type of study design				
Case–control study	10	0.73 (0.60–0.88)	58.30%	0.010
Cohort study	3	0.92 (0.85–1.00)	0.00%	0.598
Whether the results were adjusted for parity or not				
Yes	10	0.76 (0.63–0.93)	80.00%	<0.001
No	3	0.82 (0.61–1.11)	0.00%	0.617
Whether the results were adjusted for the use of OC or not				
Yes	7	0.81 (0.63–1.03)	76.90%	<0.001
No	6	0.66 (0.59–0.74)	0.00%	0.675
Whether the results were adjusted for tubal ligation or not				
Yes	5	0.74 (0.58–0.94)	72.20%	0.006
No	8	0.81 (0.62–1.04)	63.30%	0.008

RR (95% CI) represent the relative risk (95% CI) of epithelial ovarian cancer for the highest versus the lowest stratification of ALB.

### Meta-regression

The results of multivariable meta-regression showed that publication year (*P*=0.401), continent where the study was conducted (*P*=0.900), the type of study design (*P*=0.280), whether or not the results were adjusted for parity (*P*=0.831), the use of OC (*P*=0.580) and tubal ligation (*P*=0.655) had no significant impact on the heterogeneity.

### Sensitive analysis

Leave-One-Out sensitivity analysis was performed to evaluate the key studies that had substantial impacts on between-study heterogeneity. Two studies [3,29] were found to contribute to between-study heterogeneity. After excluding the two studies, the heterogeneity decreased to 0.0% (*P*_for heterogeneity_=0.680) and the result was still significant 0.67 (95% CI 0.61–0.73).

### Influence analysis and publication bias

The result of influence analysis showed that no study had excessive influence on the pooled RR of epithelial ovarian cancer for the highest versus the lowest stratification of ALB. No evidence of significant publication bias was found by the visual inspection of the funnel plot (Figure 4) and Egger’s test (*P*=0.581).

**Figure 4:** Funnel plot with pseudo 95% confidence limits for the analysis of ALB and risk of epithelial ovarian cancer The RR (95% CI) in every article is the RR (95% CI) of epithelial ovarian cancer for the highest versus the lowest stratification of ALB.

## Discussion

This meta-analysis assessed the association between ALB and epithelial ovarian cancer. Findings from our study provided evidence of a negative association between ALB and the risk of epithelial ovarian cancer. In the subgroup analysis, the significantly negative associations between ALB and epithelial ovarian cancer were observed in studies conducted in North America, studies with adjustment for parity, studies with adjustment for tubal ligation and case–control studies, respectively. In dose–response analysis, the risk of epithelial ovarian cancer decreased nonlinearly with the increase of ALB. We did not find a statistically significant association between ALB and epithelial ovarian cancer by different histological types, although the point estimates suggested a reduction in risk. This may be in part due to the limited number of studies with data for tumor subtypes.

The protective effect of ALB on epithelial ovarian cancer is closely related to the changes during pregnancy, and the changes include the cessation of ovulation cycle, the decrease of gonadotropin and estrogen level as well as the increase of progesterone level. During the ovulatory cycle, the repeated ruptures of the ovarian epithelium accompanied by estrogen-rich environmental exposure and rapid proliferative repair suggested by ‘Incessant ovulation hypothesis’ and the increase of inflammatory response suggested by ‘Inflammation hypothesis’ can increase the possibility of ovarian epithelial cell malignant transformation [50,51]. The ‘Gonadotropin hypothesis’ hold that the excessive gonadotropin and estrogen secretion may contribute to the deterioration of ovarian epithelial cells [52]. Thus, any factors (such as pregnancy) that reduce the number of ovulation cycle or the level of gonadotropin can lower the risk of epithelial ovarian cancer. However, these hypotheses are insufficient to explain the phenomenon that the later a woman has her last child, the lower her ovarian cancer risk is. A less well-recognized theory, the ‘ovarian clearance hypothesis’ suggests that the precancerous cells can be cleared by apoptosis under the action of elevated progesterone level during pregnancy [21,53–55]. On average, women with older ALB have more deteriorating ovarian epithelial cells than women with younger ALB. Thus the high levels of hormones during pregnancy may provide a greater benefit for women who have their last birth at an older age, in terms of reducing the risk of epithelial ovarian cancer [25,56].

Between-study heterogeneity is common in meta-analyses [57], and it is essential to explore the sources of between-study heterogeneity. In this meta-analysis, high between-study heterogeneity with *I*^2^ = 73.90% was found. Thus, we used the REM that considered both within-study and between-study variation to calculate the pooled RRs with 95% CIs. Beyond that, we also conducted a Leave-One-Out sensitivity analysis to reduce the heterogeneity. Two studies [3,29] were found to contribute to this high between-study heterogeneity. After excluding them, the heterogeneity reduced to 0.0% and the result remains significant, which suggested that our results were stable and credible. But the meta-regression with the covariates of study design, publication year, continent where the study was conducted, whether or not the results were adjusted for parity, the use of OC and tubal ligation failed to explain the source of heterogeneity. It indicated that some other unknown confounding factors existed in the studies.

There were many advantages in our study. First, most of the studies included in this meta-analysis had adjusted for the potential confounders that had a greater impact on the association between ALB and epithelial ovarian cancer (such as parity and tubal ligation). Second, the reverse association between ALB and epithelial ovarian cancer had no substantial change in the sensitivity analysis, which might suggest that the results were reasonable and convincing. Finally, we further conducted a dose–response analysis to explore the association between ALB and epithelial ovarian cancer.

However, several potential limitations in our study should also be considered. First, some studies including participants who were pre-menopausal might have a risk of reverse causality. Women who had epithelial ovarian cancer at a younger age might have their ovaries removed, and so would not be able to have children at an older age. This might confound the protective effect of a later ALB on epithelial ovarian cancer. Second, the age range at baseline of participant varied in every study. Finally, the adjustment factors were different among studies, and residual confounding could not be eliminated thoroughly.

## Conclusion

In summary, results from this meta-analysis indicated that ALB was negatively associated with epithelial ovarian cancer. The results mainly came from case–control studies, and thus more cohort studies were needed to confirm the conclusion.

## Abbreviations

ALB: age at last birth
CI: confidence interval
OC: oral contraceptive
REM: random-effect model
RR: relative risk
